RETRACTED

# Effects of microRNA-146a on the proliferation and apoptosis of human osteoarthritis chondrocytes by targeting *TRAF6* through the NF-κB signalling pathway

**DOI:** 10.1042/BSR20160578

**Published:** 2017-04-28

**Authors:** Jun-Hua Zhong, Jing Li, Cui-Fang Liu, Ning Liu, Rui-Xiang Bian, Shou-Mei Zhao, Shu-Yi Yan, Yong-Bing Zhang

**Affiliations:** 1 Department of Surgery, Dongying People’s Hospital, Dongying 257091, P.R. China; 2 Department of Joint Surgery, Dongying People’s Hospital, Dongying 257091, P.R. China

**Keywords:** Chondrocyte, MicroRNA-146a, NF-κB signaling pathway, Osteoarthritis, Proliferation, TRAF6

## Abstract

The present study aims to investigate the effects of *miR-146a* on the proliferation and apoptosis of human osteoarthritis (OA) chondrocytes by targeting tumour necrosis factor receptor-associated factor 6 (TRAF6) through nuclear factor-κB (NF-κB) signalling pathway. Human normal and OA chondrocytes were selected and divided into the normal group, blank group, negative control (NC) group, *miR-146a* mimics group, *miR-146a* inhibitors, *miR-146a* inhibitor + si-TRAF6 group and si-TRAF6 group. Quantitative real-time PCR (qRT-PCR) was applied to detect the expressions of *miR-146a*, *TRAF6* mRNA and *NF-κB* mRNA. Western blotting was used to detect the protein expressions of TRAF6 and NF-κB. CCK-8 assay and flow cytometry were used to detect cell proliferation and apoptosis. Compared with normal chondrocytes, the expression of *miR-146a* decreased, while the mRNA and protein expressions of TRAF6 and NF-κB increased in OA chondrocytes. OA chondrocytes had a lower proliferation rate and a higher apoptosis rate than the normal chondrocytes. Compared with the blank, NC and si-TRAF6 groups, the expression of *miR-146a* increased in the *miR-146a* mimics group, but decreased in the *miR-146a* inhibitors and *miR-146a* inhibitor + si-TRAF6 groups. Compared with the blank, NC and *miR-146a* inhibitor + si-TRAF6 groups, the mRNA and protein expressions of TRAF6 and NF-κB decreased, cell proliferation rate increased and cell apoptosis rate decreased in the *miR-146a* mimics and si-TRAF6 groups, while opposite trends were observed in the *miR-146a* inhibitors group. Our study suggests that *miR-146a* could promote proliferation and inhibit apoptosis of OA chondrocytes by inhibiting TRAF6 expression and suppressing the activation of NF-κB signalling pathway.

## Introduction

Osteoarthritis (OA) is a degenerative disease in the joints, biochemically characterized by uncontrolled destruction of cartilage matrix, new bone formation at the joint margins (osteophytes), limited inflammation (synovitis) and changes in subchondral bone structure (sclerosis) [1]. Due to increasing prevalence of obesity and an aging population, OA has become an increased worldwide health burden, leading to unbearable pain and even disability [2]. It is believed that OA results from a complex interaction between systematic factors and local factors, including age, sex, obesity, genetics and so on [3]. An increasing number of clinical studies have implied the importance of genes during the progression of OA [4,5].

miRNAs are endogenous small non-coding RNAs (approximately 22 nts long), which can regulate gene expression post-transcriptionally and have been implicated in various diseases as well as considered as potential biomarkers [6]. It is known that miRNAs play an important role in mediating the effects of the main risk factors for OA, such as aging and inflammation, through control of target genes [7–9]. The miRNAs, capable of fine tuning gene expression, are involved in the cartilage homoeostasis and thereby participated in OA pathogenesis [9]. *miR-146a* is one of the miRNAs associated with OA cartilage [10]. Previous studies have suggested *miR-146a* closely correlated with pain-related pathophysiology of OA [11,12]. An experimental study demonstrated that the expression of *miR-146a* was lower in OA cartilage and its expression was induced by IL-1β stimulation [13]. *miR-146a* has a negative effect on inflammatory responses by suppressing cytokine-induced expression of interleukin-1 receptor-associated kinase-1 (IRAK1) and tumour necrosis factor receptor-associated factor 6 (TRAF6) via impairing nuclear factor-κB (NF-κB) activity and inhibiting the expression of target genes [10]. On this ground, we hypothesize that *miR-146a* may have correlations with TRAF6 and NF-κB signalling pathway in OA.

RETRACTED

To validate our hypothesis, in the present study, we obtained human articular cartilage tissues from OA patients and patients with lower extremity amputation, and human OA and normal chondrocytes were isolated from these tissues, in order to investigate the effects of *miR-146a* on the proliferation and apoptosis of human OA chondrocytes by targeting TRAF6 through NF-κB signalling pathway.

## Materials and methods

### Ethics statement

The present study was approved by the Ethics Committee of *Dongying People’s Hospital*. All patients signed informed consent in written form. The present study also complied with the guidelines and principles of the Declaration of Helsinki [14].

### Cell isolation, culture and identification

Articular cartilage tissues were obtained from OA patients with knee/hip replacement and lower extremity amputation by accident (without OA history, normal articular cartilage tissues were obtained during the operation). The samples were placed in aseptic plates containing PBS with penicillin sodium and streptomycin (1 × 10^10^ U/l) and brought to a clean bench. Cartilage tissues in articular surface were cut and abandoned using a surgical blade thin layer to avoid thin layer of fibrous cartilage on osteophytes surface. Cartilage sheets in joint-centre region were cut and taken using a surgical blade thin layer in avoidance of subchondral bone tissues. The samples were washed with 10 ml PBS containing double antibodies (1 × 10^10^ U/l) three times and then dissected into pieces (1 mm^3^) using ophthalmic scissors. The samples was added with 3 ml 0.05% collagenase II (prepared with DMEM supplemented with 10% FBS) and digested in a CO_2_ incubator at 37°C for 30 min. After blown and beaten lightly, the samples were centrifuged at 800 rev/min for 3 min. The supernatant was abandoned. Subsequently, the samples were added with 5 ml 0.2% collagenase II and digested in a CO_2_ incubator at 37°C for 8–10 h, with oscillation in every other hour. Turbid cell suspension was collected and filtered using a 120-mesh nylon screen. The clustered cells were beaten thoroughly. Then the samples were centrifuged at 1000 rev/min for 10 min and resuspended with PBS in triplicates. Finally, the samples were resuspended using DMEM and counted. The samples (2.5 × 10^4^/cm^2^) were monolayer cultured under routine conditions in a culture dish. The medium was changed after 48 h and non-adherent cells were removed. The passage cells were obtained and identified using Toluidine Blue staining. These experiments were repeated three times.

RETRACTED

### Cell grouping

Human OA and normal chondrocytes in the logarithmic growth phase were collected and divided into seven groups: the normal group (normal chondrocytes), the blank group (OA chondrocytes without any transfection), the NC group (OA chondrocytes transfected with nonsense sequences), the *miR-146a* mimics group (OA chondrocytes transiently transfected with *miR-146a* mimics plasmid), the *miR-146a* inhibitors group (OA chondrocytes transiently transfected with *miR-146a* inhibitors plasmid), the *miR-146a* inhibitor + si-*TRAF6* group (OA chondrocytes transfected with miR-146a inhibitors plasmid and *TRAF6* siRNA sequences) and the si-*TRAF6* group (OA chondrocytes transfected with *TRAF6* siRNA sequences). *TRAF6* siRNA, *miR-146a* mimics, *miR-146a* inhibitors and small RNA molecules (negative control (NC)) were synthesized by Life Technologies. *miR-146a* mimics, inhibitors and 3 μl NC diluted to 20 μmol/l were then diluted to 150 μl in the serum-free medium (SFM) and mixed with 150 μl Lipofectamine 2000 (Invitrogen Inc., Carlsbad, CA, U.S.A.). The third-generation cells in the logarithmic growth phase were inoculated in six-well plates with 1 × 10^5^ cells per well, which were cultured in normal medium containing 2 ml serum without antibiotics. Cells were transfected to 150 μl and final concentration was 50 nmol/l when cell fusion reached approximately 60–70%. The total RNA was isolated at 24 h after transfection for further studies.

RETRACTED

### Dual-luciferase reporter gene assay

Target gene analysis was preformed through a biological prediction website (http://www.microRNA.org) to determine whether *TRAF6* is a direct target gene of *miR-146a.*The full-length *TRAF6* gene 3′-UTR region was cloned and amplified. PCR products were cloned into multiple cloning sites of a luciferase downstream gene in a pmirGLO vector (Promega Corp., Madison, WI, U.S.A.). The predicted binding site of *miR-146a* and its target gene were subjected to site-specific mutagenesis. *Renilla* luciferase-expressing pRL-TK vectors (TaKaRa) were used as an internal control to adjust for differences in cell numbers and transfection efficiency. *miR-146a* mimics and negative NC were transfected into chondrocytes with luciferase vectors respectively. The dual-luciferase reporter gene assay was performed according to the instructions of Promega Company. These experiments were repeated three times.

### Quantitative real-time polymerase chain reaction

Following the isolation of total RNA with TRIzol, RNA purification and concentration were measured with UV spectrophotometry and RNA integrity was tested by agarose gel electrophoresis. Reverse transcription was conducted with Primescript™ RT reagent kit (Takara Biotechnology Ltd., Dalian, China). PCR amplification was performed with SYBR® premix Ex Taq™ kit (Takara Biotechnology Ltd., Dalian, China). All the PCR sequences were presented in Table 1. Opticon Monitor 3 software (Bio–Rad, Inc., Hercules, CA, U.S.A.) was used to analyse the results of PCR. For calculation of the threshold cycle (*C*_t_), the threshold value was manually set as the lowest point of the raising-in-parallel logarithmic amplification circuits. Data analysis was conducted with 2^−ΔΔ*C*^_t_ method (ΔΔ*C*_t_ = (*C*_t__(target gene)_ – *C*_t__(control gene)_) _experiment group_ – (*C*_t__(target gene)_ – *C*_t__(control gene)_) _control group_). The assay was conducted in triplicates.

**Table 1:** PCR primers sequences of *miR-146a*, U6, TRAF6, NF-κB and GAPDH

Gene	Sequence
*miR-146a*	
Upstream primer	5′-TGAGAACTGAATTCCATGGGTT-3′
Downstream primer	5′-CCCAUGGAAUUCAGUUCUCAUU-3′
*U6*	
Upstream primer	5′-CTCGCTTCGGCAGCACA-3′
Downstream primer	5′-ACGCTTCACGAATTTGCGT-3′
*TRAF6*	
Upstream primer	5′-TTCATAGCTTGAGCGTTATACCCGAC-3′
Downstream primer	5′-CAGACTGATCAAGAATTGTAAGGCGTA-3′
*NF-κB*	
Upstream primer	5′-CTGAACCAGGGCATACCTGT -3′
Downstream primer	5′-GAGAAGTCCATGTCCGCAAT -3′
*GAPDH*	
Upstream primer	5′-AGAAGGCTGGGGCTCATTTG-3′
Downstream primer	5′-AGGGGCCACAGTCTTC-3′

GAPDH, glyceraldehyde phosphate dehydrogenase.

RETRACTED

### Western blotting

Transfected chondrocytes were washed with PBS twice and were lysed in 100 μl lysis solution at 4°C for 30 min. Then the samples were centrifuged (12000 rev/min) for 10 min and the supernatant was collected. Protein concentration was determined with Bradford assay. The samples (50 μg protein/lane) underwent SDS/PAGE and were electrotransferred into a PVDF membrane. The membrane was blocked with 5% skimmed milk at room temperature for 1 h and incubated overnight at 4°C with primary antibodies (Abcam Inc., Cambridge, MA, U.S.A.), including TRAF6 (EP592Y, 1:5000 dilution), NF-κB (E379, 1:50000 dilution) and GAPDF (ab9485, 1:2500 dilution). Subsequently, the membrane was washed and incubated with secondary antibody horseradish peroxidase (HRP) at room temperature in light-proof environment for 1 h. Then the membrane was rinsed thoroughly and imaged with an Odssey dual-color infrared laser imaging system. Integrated optical density of each band was calculated. The relative expression of target protein was calculated as the ratio between integrated optical density of target bands and that of GAPDH bands (internal control bands). These experiments were repeated three times.

### CCK-8 assay

After digestion and centrifugation, cells (1 × 10^4^ cells/well) were seeded into 96-well plates with six repeated wells in each group. Cells were transfected after 24 h and then incubated with complete medium for 4–6 h after transfection. At 0, 12, 24 and 48 h after transfection, culture medium was removed. Then transfected cells were incubated with evenly blending and bubble-free mixture of WST (10 μl) and DMEM (90 μl) medium at 37°C with 5% CO_2_ for 2 h. Subsequently, the optical density (OD) was detected at 450 nm (650 nm as reference) using a microplate reader. These experiments were repeated three times.

### Flow cytometry

After digestion and centrifugation, cells (1 × 10^5^ cells/well) were seeded into six-well plates with conventional transfection. At 48 h after transfection, cells were digested by 0.25% EDTA-free trypsin. To avoid cell damage by overdigestion, a microscope was used to keep close observation. Approximately 2–3 min later, when most cells rounded up, the digestion was ended using complete medium. The cell suspension was moved to EP tubes. Cells were rinsed with PBS twice, centrifuged at 1500 rev/min for 5 min and resuspended in 500 μl binding buffer. One microlitre Annexin V-PE (Annexin V-Phycoerythrin) and 5 μl 7-AAD (7-Aminoactinomycin D) were added and mixed. The reaction was incubated for 10 min. Cell apoptosis was detected by a flow cytometry within 1 h. These experiments were repeated three times.

RETRACTED

### Statistical analysis

Data were analysed using SPSS 21.0 software (SPSS Inc., Chicago, IL, U.S.A.). Categorical data were expressed with frequency or percentage. Chi-square test was applied for between-group comparison. Numerical data were described as mean ± S.D. The *t* test was applied for pairwise comparison of the mean value. After homogeneity test of variance, one-way ANOVA was used for multigroup comparison. Least significant difference (LSD) *t* test was used for pairwise comparison of the mean value among groups. Two-tailed *P*<0.05 was considered statistically significant.

## Results

### Identification of human normal and OA chondrocytes

Under an inverted microscope, human normal primary chondrocytes were adherent at 24 h after inoculation. Most adherent chondrocytes were round, oval or short spindle-shaped with abundant cytoplasm. The nuclei were round and centred with 1–3 nucleolus in uniform dispersion, like a smiling face. Some cells showed confluent growth like cobblestones. The cells were covered the bottom of culture bottle and up to 80% after approximately 14 days. OA chondrocytes were adherent at 24–28 h after inoculation. Most adherent chondrocytes were long spindle-shaped, irregular or dendritic, like cobblestones. Cell colonies were rare with a slower growth. The primary chondrocytes covered the bottom of culture bottle and up to 80% after 20 days. Toluidine Blue staining was applied for identification of normal chondrocytes and OA chondrocytes. Blue-purple metachromatic granules could be seen in both of them. Nuclei and cytoplasm were stained dark blue and light blue respectively. Human normal chondrocytes were regular and larger, with more blue-purple metachromatic granules (Figure 1A). However, OA chondrocytes were irregular and smaller, with less blue-purple metachromatic granules (Figure 1B).

**Figure 1:** Toluidine Blue staining of human normal and OA chondrocytes (×200) (**A**) Normal chondrocyte; (**B**) OA chondrocytes.

### Targeting relationship between *miR-146a* and *TRAF6*

Biological prediction website (microRNA.org) presented that *miR-146a* could target *TARF6* (Figure 2A). To validate this finding, *TRAF6* mRNA 3′-UTR was inserted to luciferase reporter vectors to construct recombinant plasmids, pTRAF6 wild-type (pTRAF6-WT) and *pTRAF6* mutant type (pTRAF6-MT). Compared with the *TRAF6* 3′-UTR-WT + NC, *TRAF6* 3′-UTR-MT + NC and *TRAF6* 3′-UTR-MT + *miR-146a* mimics groups, fluorescence signal decreased approximately 44% in the *TRAF6* 3′-UTR-WT + mimics group (*P*<0.05). There was no significant difference in fluorescence signal between the *TRAF6* 3′-UTR-MT + NC and *TRAF6* 3′-UTR-MT + *miR-146a* mimics groups (*P*>0.05) (Figure 2B). Therefore, we believed that *TRAF6* is a target gene of *miR-146a* and *miR-146a* could target and regulate *TRAF6* mRNA*.*

RETRACTED

**Figure 2:** Verification of targeting relationship between *miR-146a* and TRAF6 (**A**) microRNA.org for detection of *miR-146a* targeting *TRAF6*; (**B**) dual-luciferase reporter gene assay; * refers to *P*<0.05 compared with WT + mimics.

### *miR-146a* expressions in human normal and OA chondrocytes

The results of quantitative real-time PCR (qRT-PCR) demonstrated that compared with the normal group, *miR-146a* expression decreased in the blank, NC, *miR-146a* mimics,* miR-146a* inhibitors, *miR-146a* inhibitor + si-TRAF6 and si-TRAF6 groups. Compared with the blank group, *miR-146a* expression increased in the *miR-146a* mimics group, but decreased in the *miR-146a* inhibitors and *miR-146a* inhibitor + si-TRAF6 groups (all *P*<0.05). No significant difference was observed among the NC, si-TRAF6 and blank groups (*P*>0.05) (Figure 3).

**Figure 3:** The expressions of miR-*146a* in human normal and OA chondrocyte * refers to *P*<0.05 compared with the normal group; ^#^ refers to *P*<0.05 compared with the blank group; *n*=3.

### The mRNA expressions of TRAF6 and NF-κB in human normal and OA chondrocytes

The results of qRT-PCR indicated that compared with the normal group, the mRNA expressions of *TRAF6* and NF-κB incresed in the blank, NC, *miR-146a* mimics, *miR-146a* inhibitors, *miR-146a* inhibitor + si-TRAF6 and si-TRAF6 groups. Compared with the blank group, the mRNA expressions of *TRAF6* and NF-κB decreased in the *miR-146a* mimics and si-TRAF6 groups, but increased in the *miR-146a* inhibitors group (all *P*<0.05). There was no significant difference among the NC, *miR-146a* inhibitor + si-TRAF6 and blank groups (*P*>0.05) (Figure 4).

**Figure 4:** The mRNA expressions of *TRAF6* and *NF-κB* in human normal and OA chondrocytes * refers to *P*<0.05 compared with the normal group; ^#^ refers to *P*<0.05 compared with the blank group; *n*=3.

### The protein expressions of TRAF6 and NF-κB in human normal and OA chondrocytes

The results of Western blotting showed that compared with the normal group, the protein expressions of *TRAF6* and NF-κB incresed in the blank, NC, *miR-146a* mimics, *miR-146a* inhibitors, *miR-146a* inhibitor + si-TRAF6 and si-TRAF6 groups. Compared with the blank group, the protein expressions of *TRAF6* and NF-κB decreased in the *miR-146a* mimics and si-TRAF6 groups, but increased in the *miR-146a* inhibitors group (all *P*<0.05). No significant difference was exhibited among the NC, *miR-146a* inhibitor + si-TRAF6 and blank groups (*P*>0.05) (Figure 5).

RETRACTED

**Figure 5:** The protein expressions of TRAF6 and NF-κB in human normal and OA chondrocytes (**A**) Protein expressions; (**B**) protein bands; * refers to *P*<0.05 compared with the normal group; ^#^ refers to *P*<0.05 compared with the blank group; *n*=3.

### Cell proliferation of human normal and OA chondrocytes

The results of CCK-8 presented that compared with the normal group; cell growth was slower in the blank, NC, *miR-146a* mimics, *miR-146a* inhibitors, *miR-146a* inhibitor + si-*TRAF6* and si-*TRAF6* groups. Compared with the blank group, cell growth was faster in the *miR-146a* mimics and si-TRAF6 groups, but was slower in the miR-146a inhibitors group (*P*<0.05). There was no significant difference among the NC, *miR-146a* inhibitor + si-TRAF6 and blank groups (*P*>0.05) (Figure 6).

**Figure 6:** Cell proliferation of human normal and OA chondrocytes * refers to *P*<0.05 compared with the normal group; ^#^ refers to *P*<0.05 compared with the blank group; *n*=3.

### Cell apoptosis of human normal and OA chondrocytes

The results of flow cytometry revealed that compared with the normal group; cell apoptosis rate increased in the blank, NC, *miR-146a* mimics, *miR-146a* inhibitors, *miR-146a* inhibitor + si-*TRAF6* and si-TRAF6 groups. Compared with the blank group, apoptosis rate decreased in the *miR-146a* mimics and si-TRAF6 groups, but increased in the *miR-146a* inhibitors group (*P*<0.05). No significant difference was observed among the NC, *miR-146a* inhibitor + si-TRAF6 and blank groups (*P*>0.05) (Figure 7).

**Figure 7:** Cell apoptosis of human normal and OA chondrocytes * refers to *P*<0.05 compared with the normal group; ^#^ refers to *P*<0.05 compared with the blank group; *n=*3.

## Discussion

Serveral studies have demonstrated that up-regulation of *miR-146a* expression may be an effective strategy for the treatment of inflammatory arthritis [9,15–17]. Evidence suggested that *miR-146a* could inhibit the expressions of IRAK1 and *TRAF6*, impair NF-κB signalling pathway and suppress NF-κB-related gene expressions [13,16–18]. Transfection with synthetic *miR-146a* could suppress extracellular matrix related proteins in chondrocytes and inhibit inflammatory cytokines in synovial cells obtained from human knee joints [11]. In the present study, the effects of* miR-146a* on the proliferation and apoptosis of human OA chondrocytes by targeting TRAF6 through NF-κB signalling pathway were investigated.

RETRACTED

Through information collection from relevant website and a dual-luciferase reporter gene assay, we first verified the association between *miR-146a* and *TRAF6*. *miR-146a* could target *TRAF6* in the *TRAF6*-3′-UTR region. We also found that the mRNA expression of *TRAF6* and NF-κB decreased in the *miR-146a* mimics group while increased in the *miR-146a* inhibitors group. Thus, we preliminarily considered that *miR-146a* had a negative association with *TRAF6* and NF-κB. Concordantly, we also observed that the protein expressions of *TRAF6* and NF-κB decreased in the *miR-146a* mimic group while increased in the *miR-146a* inhibitors group. Based on the above results, we felt safe to conclude that *miR-146a* could inhibit the mRNA and protein expressions of *TRAF6* and NF-κB in OA. Li et al. [11] revealed a significant correlation between arthritic joint pathogenesis and *miR-146a*, indicating that *miR-146a* regulated cartilage-degrading proteases and pain associated inflammatory molecules in the peripheral knee joint tissues including articular chondrocytes and synoviocytes. In addition, *TRAF6*, a key adaptor molecule in NF-κB and TLR signalling pathways, is a direct target of *miR-146a* through a negative feedback regulation loop [19].

Our results showed that with *miR-146a* overexpression inhibiting *TRAF6*, cell proliferation was increased in the *miR-146a* and si-TRAF groups, with *miR-146a* inhibition weakening the influence of *miR-146a* on *TRAF6*, cell proliferation is decreased in the *miR-146a* inhibitors group. Therefore, we believed that *miR-146a* may positively activate cell proliferation through suppressing *TRAF6*. Chondrocyte proliferation, as a clinical feature of OA, has self-healing ability to repair joint damage [20]. In addition, our observation on cell apoptosis also suggested that *miR-146a* overexpression in the mimics group had less cell apoptosis. Recent evidence demonstrated that chondrocyte apoptosis is a potential target to protect articular cartilage in OA [21]. Several studies have indicated that the cell apoptosis rate of chondrocytes is increased in OA cartilage and have authenticated the role of apoptosis in the pathogenesis of OA [22–24]. In this context, we believed that *TRAF6*-mediating *miR-146a* may be a potential therapeutic target. Prior to our study, researchers also reported that through inhibition of SMAD4, increased *miR-146a* could promote transforming growth factor β (TGF-β) induced cell proliferation and reduce cell apoptosis in cancers [25,26].

## Conclusion

In conclusion, we provided strong evidence that *miR-146a* could target *TRAF6* through NF-κB signalling pathway and negatively regulate their mRNA expressions and protein expressions in OA. Besides, *miR-146a* could influence cell proliferation and apoptosis of chondrocytes possibly through regulation of *TRAF6*. In a word, *miR-146a* targeting *TRAF6* through NF-κB signalling pathway may be a potential therapeutic target for OA. However, we only looked at TRAF6, while we did not choose other targets of *miR-146a* that were involved in NF-κB regulation, which might affect the reliability of our results.

RETRACTED

## Abbreviations

CCK-8: cell counting kit-8
*C*_t_: threshold cycle
EP: eppendorf
GAPDH: glyceraldehyde phosphate dehydrogenase
IRAK1: interleukin-1 receptor-associated kinase-1
IL-1: interleukin-1β
MT: mutant type
NC: negative control
NF-κB: nuclear factor-κB
OA: osteoarthritis
qRT-PCR: quantitative real-time PCR
TRAF6: tumour necrosis factor receptor-associated factor 6
WT: wild-type
